# Surgical Treatment of Bilateral Chronic Subdural Hematoma

This article has been retracted.

**DOI:** 10.1155/2022/2823314

**Published:** 2022-06-27

**Authors:** Yan Zhuang, Ming Jiang, Jiahao Zhou, Jun Liu, Zhen Fang, Zejun Chen

**Affiliations:** Department of Neurosurgery, The Affiliated Hospital of Jiangsu University, 438 Jiefang Road, Zhenjiang 212001, Jiangsu Province, China

## Abstract

**Background:**

Chronic subdural hematoma (CSDH) is one of the common clinical intracranial hemorrhagic disorders, accounting for 16%–20% of bilateral CSDH. At present, the surgical treatment of bilateral CSDH mainly includes drilling drainage and neuroendoscopic assistance. The main objective of this paper was to compare the effects of two surgical methods on CSDH.

**Methods:**

153 patients who were diagnosed with CSDH were included in this study. 79 patients were treated with bilateral drilling drainage, and the other 74 patients were treated with neuroendoscope-assisted drainage. The clinical data of the two groups were compared, and the surgical indexes, neurological function, cure rate, and recurrence rate of the two groups were compared. The operation indexes of patients include operation time, postoperative hematoma volume, hospital stay, extubation time, misplacement of drainage tube, recurrence, and hematoma clearance rate.

**Results:**

All patients underwent CT  examination one day after operation. The CT  imaging detection of the two groups was generally good. The cranial CT was reexamined before discharge. The bilateral hematoma disappeared in 114 patients, the unilateral hematoma disappeared in 29 patients, a small amount of compensatory crescent very low-density shadow subdural effusion was observed on the other side, and a small amount of compensatory crescent very low-density shadow subdural effusion was observed on both sides in 10 patients. There was no space occupying effect and intracranial gas disappeared. Compared with neuroendoscopic assisted drainage, the operation time of drilling drainage patients was significantly shorter. The extubation time, drainage tube dislocation, recurrence rate, postoperative hematoma volume, and hematoma clearance rate of patients receiving neuroendoscopic assisted drainage were significantly better than those receiving drilling drainage. The Markwalder score and hospital stay between the two groups were not significant.

**Conclusions:**

Drilling drainage and neuroendoscopic assisted surgery have good therapeutic effects on bilateral CSDH. The operation time of drilling drainage is shorter. Neuroendoscopic assisted surgery has more advantages in extubation time, misplacement of drainage tube, recurrence, postoperative hematoma volume, and hematoma clearance rate.

## 1. Introduction

CSDH is one of the common intracranial hemorrhagic disorders [1, 2]. CSDH is common in older adults, mostly secondary to head trauma [3]. Bilateral subdural hematomas have the characteristics of severe symptoms, rapid progress, and easy deterioration and should be treated as soon as possible [4, 5]. At present, the method of bilateral synchronous drilling, drainage, and flushing is mostly used in clinic [6, 7]. Drilling drainage has good clinical effect and can effectively remove hematoma, but there was a certain rate of catheter misplacement and risk of rebleeding. The removal of hematoma and postoperative recurrence rate need to be improved [8, 9]. Neuroendoscopy has the advantages of sufficient light, clear vision, proximity, and multi-angle observation [10–12]. At present, it is widely used in all aspects of neurosurgery. Neuroendoscopic assisted drainage has been gradually applied to the surgical treatment of CSDH. However, there is no research to explore the therapeutic effect of drilling drainage and neuroendoscopic assisted drainage in patients with bilateral CSDH.

In this study, patients with bilateral CSDH were collected and treated with bilateral drilling drainage or neuroendoscope-assisted drainage to explore the therapeutic effects of the two surgical methods on patients with bilateral CSDH.

## 2. Methods

### 2.1. Patients

A total of 153 patients with bilateral CSDH were included in this study. There were 89 male patients and 64 female patients. The average age was (60.95 ± 10.26) years. All patients were clinically diagnosed with bilateral CSDH. There were 72 cases with definite history of trauma. The time from trauma to diagnosis of bilateral CSDH was 3 weeks to 3 months. There were 60 cases of hypertension and 43 cases of diabetes mellitus. Among them, 79 patients underwent bilateral drilling drainage, and 74 patients underwent neuroendoscopic assisted drainage. The neuroendoscopy group patients underwent assisted drainage through neuroendoscopy. The drilling drainage group patients underwent trans-drilling drainage. The history of trauma, the history of hematoma, and the amount of hematoma between the two groups patients were not significant (*P* < 0.05). All patients voluntarily signed the informed consent form. This study was approved by the ethics review committee of our hospital.

### 2.2. Inclusion Criteria

The patients met the diagnostic criteria of bilateral CSDH. The patients developed symptoms of chronic intracranial hypertension 3 weeks after trauma or had no definite history of trauma. Head CT showed bilateral crescent high, low, or mixed density shadows, with varying degrees of compression or midline displacement of brain tissue. MRI showed that T1 and T2 were high signals in the early stage, and T1 was slightly higher than the low signal and T2 was high signal in the later stage. Patients can undergo neuroendoscopic surgery or drilling drainage surgery.

### 2.3. Exclusion Criteria

Exclusion criteria were as follows: the patient has severe disability and basic diseases and cannot tolerate general anesthesia and endoscopic surgery; GCS score <5 or mydriasis (unilateral or bilateral); there is severe coagulation dysfunction; acute subdural hematoma; and unilateral CSDH.

### 2.4. Surgical Methods

Patients in neuroendoscopy group underwent hematoma removal under rigid neuroendoscopy under general anesthesia. The patient was in lateral or supine position, and a 4∼5 cm scalp straight incision was made on the forehead and temporal part. The mastoid process spreader was used to open, the skull was drilled, and a bone flap with a diameter of 2.5∼3 cm was formed with a milling cutter. After drilling the skull edge, suspend the dura mater, open the dura mater in the “ten” way, and try not to open the subdural hematoma capsule. We slowly aspirate part of the liquefied hematoma with a syringe to slowly reduce the intracranial pressure. After bipolar electrocoagulation and electrocautery of the hematoma capsule, cut it off, put a 30° hard neuroendoscope with a diameter of 4 mm into the subdural cavity, remove the residual hematoma under the neuroendoscope, remove the inflammatory capsule of the hematoma cavity as much as possible, and open the separation. After the hematoma is cleared, rinse with normal saline, place the drainage tube into the subdural cavity under the direct vision of neuroendoscope, carefully check that there is no bleeding in the hematoma cavity, and tightly suture the dura mater after exhausting the air with normal saline. The bone flap was returned and fixed, and the scalp was sutured in layers.

The patients in the drilling drainage group underwent drilling drainage under local anesthesia. In the supine or lateral position, make a 3∼4 cm scalp straight incision on the thickest parietal tubercle or forehead of the hematoma, open the mastoid expander, drill the skull, cut the dura mater and hematoma capsule, see the dark red bloody liquid gushing out, place the drainage tube, repeatedly lavage until the drainage fluid is clear, fix the drainage tube and suture the wound. Routine symptomatic support treatment was given after operation. CT was rechecked on the 1st day after operation and the day before discharge. If the brain tissue was satisfactory and the midline was well repositioned, the drainage tube was pulled out.

### 2.5. Observation Indexes

The surgical indexes, neurological function, cure, and recurrence of the two groups were compared. The operation indexes of patients include operation time, hospital stay, extubation time, misplacement of drainage tube, recurrence, postoperative hematoma volume, and hematoma clearance rate. Neurological function was evaluated by Markwalder classification: grade 0: normal neurological function; grade 1: clear mind, headache, and dizziness; grade 2: focal neurological dysfunction and disorientation; grade 3: severe neurological dysfunction; grade 4: loss of brain control.

### 2.6. Statistical Analysis

The data generated in this study were analyzed by SPSS 26.0 software. Measurement data are expressed as *x* ± *s*, and *t*-test is performed. The measurement data are expressed as *n* (%), and the chi-square test is performed. *P* < 0.05 indicates a significant difference.

## 3. Results

### 3.1. Comparison of Preoperative Clinical Data in Patients with Bilateral CSDH

The clinical data of patients in the neuroendoscopy group were compared with the patients from drilling drainage group (Table 1). The gender, age, history of hypertension, history of diabetes, history of trauma, midline shift, preoperative hematoma volume, and Markwalder classification between the two groups were not significant.

### 3.2. Postoperative Imaging Findings

All patients were examined by CT one day after operation. The bilateral hematoma cavities of 82 patients were almost closed, the unilateral hematoma cavities of 57 patients were almost closed, and the contralateral hematoma cavities decreased significantly. The hematoma cavity of 14 patients was significantly reduced, and the CT manifestation of the residual hematoma cavity was crescent low-density shadow under the inner plate of skull. Five patients had a small amount of intracranial pneumatosis, and there was no space occupying effect. Before the drainage tube was removed, the skull CT was rechecked, and the hematoma cavity was further reduced. The cranial CT was reexamined before discharge. Bilateral hematoma disappeared in 114 patients, unilateral hematoma disappeared in 29 patients, with a small amount of compensatory crescent very low-density shadow subdural effusion in the other side, and bilateral compensatory crescent very low-density shadow subdural effusion in 10 patients. There was no space occupying effect and intracranial gas disappeared (Figure 1).

### 3.3. Comparison of Operation Indexes of Patients

Compared with the patients in the drilling drainage group, the operation time was prolonged, the extubation time was shortened, the amount of postoperative hematoma was reduced, and the displacement of drainage tube, recurrence rate, and hematoma clearance rate were improved in the neuroendoscopy group, but there was no significant difference in hospital stay and Markwalder score (Table 2).

## 4. Discussion

CSDH is one of the common disorders in neurosurgery. The incidence of chronic subdural hematoma is on the rise as the population ages. CSDH is more common in older men with a history of mild head trauma, and the source of bleeding and pathogenesis are not fully understood [13, 14]. The traditional view is that slight head trauma causes the tear of bridging vein and a small amount of subdural bleeding. After bleeding, it is secondary to hyperfibrinolysis and the increase of local fibrin degradation products, resulting in the continuous bleeding of new capillaries and the gradual increase of hematoma [15, 16]. CSDH accounts for about 10% of all intracranial hematomas, and bilateral CSDH accounts for about 16%–20% [17–19] of all CSDH.

The recurrence rate of bilateral CSDH is high, and the clinical manifestations are changeable. Nausea and vomiting are common, and hemiplegia is rare. It is considered that bilateral hemorrhage leads to the relative balance of bilateral cerebral hemisphere compression, and the probability of midline deviation is small [20, 21]. For bilateral CSDH, some studies suggest that bilateral simultaneous decompression should be given as soon as possible, and even cases with only mild neurological deficit should be actively treated. It is proposed that MRI examination of T1 low signal and T2 high and low mixed signal indicates that it will deteriorate rapidly and need urgent surgical treatment [22–24]. In terms of treatment methods, some studies believe that there was no significant difference in complications and hospital stay between extended resection of fibrous membrane of hematoma after large bone flap craniotomy and local drilling fibrous membrane resection, but the former can reduce the recurrence of hematoma [25–27]. Some studies believe that middle meningeal artery embolization can prevent hematoma expansion and recurrence in patients with recurrence after multiple surgical treatments [28]. At present, bilateral drilling drainage is recommended for most patients with bilateral CSDH [29].

Neuroendoscopy can help identify and destroy new membranes, septa, and solid blood clots and stop bleeding under direct vision. The endoscopic monitoring system can guide the operation and avoid blind operation [30, 31]. Endoscopy can not only clearly see the shape, structure, adhesion, and separation of the capsule but also separate and open the separation of the organized adhesion in the hematoma cavity under direct vision, which greatly improves the thoroughness of hematoma removal [32–34]. Neuroendoscopy can directly stop other obvious small active bleeding in the cavity with endoscopic bipolar electrocoagulation, which reduces the incidence of postoperative rebleeding.

The results of this study showed that in the patients who received bilateral drilling drainage and neuroendoscopic assisted drainage, the bilateral hematoma cavities of most patients were almost closed one day after operation, and a small number of patients had a small amount of intracranial gas. There was no death or major complications, which showed that the effects of bilateral drilling drainage and neuroendoscopic assisted drainage were good. Compared with the patients in the drilling drainage group, the operation time was prolonged, the extubation time was shortened, the amount of postoperative hematoma was reduced, and the displacement of drainage tube, recurrence rate, and hematoma clearance rate were improved in the neuroendoscopy group, but there was no significant difference in hospital stay and Markwalder score.

The above results show that drilling drainage and neuroendoscopic assisted drainage have good therapeutic effects on patients with bilateral CSDH. Neuroendoscopy has the advantages of extubation time period, low misplacement and recurrence rate of drainage tube, low amount of postoperative hematoma and high clearance rate of hematoma. When the surgical conditions are met, the way of neuroendoscopic assisted drainage may be more conducive to the treatment and prognosis of patients with bilateral CSDH. However, due to the small sample size of this study, some results may be biased. In the later stage, we still need to collect more samples and relevant clinical indicators for more detailed research and discussion.

## Figures and Tables

**Figure 1:** Preoperative and postoperative imaging examination of patients. (a) Preoperative MRI T1 weighted imaging of a patient in neuroendoscopy group. (b) Preoperative MRI T2 weighted imaging of a patient in neuroendoscopy group. The preoperative MRI results showed that there were different degrees of hematomas on both sides of the patient's brain. (c) CT image of a patient in neuroendoscopy group one day after operation. The hematoma area of the patient decreased significantly. (d) CT images of a patient in neuroendoscopy group one day before discharge. The bilateral hematoma cavities of the patient were almost closed. (e) T1 weighted MRI of a patient in drilling drainage group before operation. (f) Preoperative MRI T2 weighted imaging of a patient in drilling drainage group. Bilateral subdural hematoma was diagnosed. (g) CT  images of one patient in drilling drainage group one day after operation. The patient's unilateral hematoma cavity was almost closed. (h) CT  image of a patient in drilling drainage group one day before discharge. The patient's bilateral hematoma cavity was almost closed.

**Table 1:** Comparison of general data between the two groups of patients.

Clinical data	Neuroendoscopy (*n* = 74)	Drilling drainage (*n* = 79)	*t/X* ^*2*^	*P*
Gender (male/female)	40/34	49/30	0.998	0.318
Age (y)	62.83 ± 9.67	61.27 ± 10.94	0.932	0.353
History of hypertension	27 (36.49)	33 (41.77)	0.448	0.503
Diabetes history	20 (27.03)	23 (29.11)	0.082	0.774
History of trauma	32 (43.24)	40 (50.63)	0.838	0.360
Midline shift	26 (35.14)	31 (39.24)	0.276	0.600
Preoperative hematoma volume (mL)	138.76 ± 20.08	143.59 ± 18.07	1.566	0.120
Markwalder	2.43 ± 0.48	2.39 ± 0.37	0.579	0.563

**Table 2:** Comparison of surgical indexes between the two groups of patients.

Clinical data	Neuroendoscopy (*n* = 74)	Drilling drainage (*n* = 79)	*t/X* ^*2*^	*P*
Operation time (min)	49.76 ± 6.08	34.67 ± 5.23	16.490	0.000
Hospital stay (d)	14.65 ± 1.79	14.16 ± 1.83	1.673	0.097
Extubation time (d)	4.21 ± 0.85	5.76 ± 0.94	10.670	0.000
Misplacement of drainage tube	0 (0.00)	6 (7.59)	5.850	0.016
Recrudescence	1 (1.35)	7 (8.86)	4.348	0.037
Postoperative hematoma volume (mL)	21.64 ± 4.67	45.08 ± 6.72	24.900	0.000
Hematoma clearance rate	89.64 ± 7.18	74.95 ± 8.67	11.370	0.000
Markwalder	0.86 ± 0.09	0.83 ± 0.11	1.839	0.068

## Data Availability

No data were used to support this study.
